The article "Blood Parameter Profiles and Their Clinical Implications in Hypertensive Patients: A Retrospective Chart Review" was retracted in 2025. Reasons: errors in the data; errors in the methods; errors in the results or conclusions; errors in the images.

# Blood Parameter Profiles and Their Clinical Implications in Hypertensive Patients: A Retrospective Chart Review

**DOI:** 10.7759/cureus.43691

**Published:** 2023-08-18

**Authors:** Ahmed S Al Zomia, Zia Sabah, Mosab Deajim, Abdullah H Alamri, Ghufran B Asiri, Lama A Lahiq, Wajd Alhadi, Nasser A Alwaqdi

**Affiliations:** 1 College of Medicine, King Khalid University, Abha, SAU; 2 Department of Medicine, King Khalid University, Abha, SAU; 3 Department of Medicine and Surgery, King Khalid University, Abha, SAU

**Keywords:** saudi arabia, electrolyte balance, creatinine, hemoglobin, hematological parameters, hypertensive patients

## Abstract

Introduction

Hypertension (HTN) is a chronic condition that serves as a major risk factor for cardiovascular diseases, leading to increased mortality and morbidity. It is a frequent modifiable illness affecting global health, resulting in catastrophic fatalities and morbidity.

Aim

This study aims to investigate blood parameter profiles and their clinical implications in hypertensive patients at the Prince Faisal bin Khalid Cardiac Center in Abha, Saudi Arabia.

Methods

Utilizing retrospective data from 121 patients at the Prince Faisal bin Khalid Cardiac Center in Abha, Saudi Arabia. The hematological parameter examined were hemoglobin (HB), platelets, hematocrit (HCT), calcium, phosphorus, sodium, potassium, urea, creatinine, and uric acid. The SPSS version 28 software was used for data analysis.

Results

Significant correlations between various hematological parameters were found in the results, pointing to potential connections between kidney function, the production of blood cells, and electrolyte balance in hypertensive patients. The results align with earlier studies carried out in the area and offer insightful information for clinicians and researchers interested in managing HTN and its complications.

Conclusion

The study emphasized the significance of considering hypertensive patients' age, gender, and lifestyle when interpreting their blood parameter profiles. The findings imply that a thorough comprehension of these blood parameter values and their potential effects on HTN is necessary for effectively managing HTN in this population. This study on the blood parameter profiles in hypertensive patients in Saudi Arabia provides the relationships between various hematological parameter and their clinical implications. These findings should be considered when creating targeted interventions and strategies to address the specific requirements and difficulties of managing HTN and its associated complications in this population. More research is required to comprehend the underlying reasons for the observed variations in hematological parameter profiles and their effects on the management of HTN.

The article "Blood Parameter Profiles and Their Clinical Implications in Hypertensive Patients: A Retrospective Chart Review" was retracted in 2025. Reasons: errors in the data; errors in the methods; errors in the results or conclusions; errors in the images.

## Introduction

Hypertension (HTN) is a frequent controllable condition that affects the worldwide population's health and causes morbidity and mortality. A total of 19.60 million hypertensive heart disease cases were documented in 2019 compared to 7.82 million in 1990, corresponding to an estimated annual percentage change of 0.17 [1]. HTN raises the risk of various conditions, including cardiovascular, metabolic, and renal illness. Furthermore, HTN has been shown to be associated with cardiovascular and musculoskeletal diseases such as osteoarthritis [2]. The prevalence of HTN varies according to geography, nation, and research sample. As a result of its high direct and indirect costs, HTN has a substantial influence on the global economy. In 2019, the prevalence of age-standardized HTN was at its lowest in Canada and Peru for both men and women. It was also notably low for women in Taiwan, South Korea, Japan, and certain Western European countries like Switzerland, Spain, and the UK. On the other hand, for men, the lowest prevalence was observed in several low-income and middle-income countries, including Eritrea, Bangladesh, Ethiopia, and the Solomon Islands [3]. The burden of HTN in persons and healthcare systems is rather high because of the increasing need for health consultations, hospitalization, laboratory and radiographic tests, and the extensive use of prescription and nonprescription medicines [4]. The diagnostic criteria for HTN have recently been updated by Hypertension Guideline Writing Committee: 130 mm Hg or higher systolic pressure and/or 80 mm Hg or higher diastolic pressure [5]. Due to urbanization, physical inactivity, and poor diet, the prevalence of HTN is anticipated to rise both regionally and internationally [6]. Previous estimates have placed the prevalence of HTN in the Saudi population at 4.9% in Al-Kharj town [7] and 15.2% in the general population across Saudi Arabia [8]. Over the last decade, the prevalence has risen from 8.9% in some areas to 15.2% in others. This rise might be attributed to a variety of demographic and economic causes [8]. Alenazi AM and Alqahtani BA investigated the national and regional incidence of HTN in the Saudi population in 2023. The prevalence of HTN in the Saudi population aged 15 and up was 9.2%. It was greater in women (10.0%) than in males (8.5%). HTN prevalence increased with age (65 and over), accounting for 55.3% in women and 48.0% in men. It was comparably low in the younger age group, accounting for 0.1% in those aged 15-19. The frequency of HTN varied greatly amongst locations, ranging from 6.0% in the Najran region to 10.0% in the Makkah region [9]. Few studies have examined hematological parameter profiles and their clinical implications in hypertensive patients. As a result, the current research was designed to investigate the relationship between HTN and hematological parameter profiles.

The article "Blood Parameter Profiles and Their Clinical Implications in Hypertensive Patients: A Retrospective Chart Review" was retracted in 2025. Reasons: errors in the data; errors in the methods; errors in the results or conclusions; errors in the images.

## Materials and methods

This is a retrospective study conducted at Prince Faisal Bin Khalid Cardiac Center located in Abha, Saudi Arabia, approximately 1.2 km from the central part of Abha. The Prince Faisal Bin Khalid Cardiac Center is a renowned medical facility that specializes in providing advanced cardiac care and treatment to patients with various heart-related conditions.

Inclusion criteria

This study encompassed all eligible hypertensive patients attending Prince Faisal Bin Khalid Cardiac Center between 2021 and 2022, aged 20 years or above, who agreed to participate in the study. 

Exclusion criteria

We excluded patients aged below 20 years and above 70 years, individuals on lipid-lowering medications, those with thyroid disease, and those with pre-eclampsia/eclampsia. Additionally, patients with hematologic derangements and hypertensive patients with co-morbid diabetes mellitus were precluded from the study to mitigate potential confounding factors.

In this study, we investigated the correlation between HTN and various laboratory parameters, including lipid profiles such as serum total cholesterol (TC), triglycerides (TGs), high-density lipoprotein cholesterol (HDL-C), and low-density lipoprotein cholesterol (LDL-C). We also examined hematologic parameters such as hemoglobin, hematocrit, RBC count, platelet count, and RBC indices. Other considered laboratory parameters included calcium, phosphorus, sodium, potassium, urea, creatinine, and uric acid. Beyond these laboratory variables, we incorporated sociodemographic factors, anthropometric measurements, and clinical characteristics to evaluate their potential impact on HTN.

Operational definitions

Dyslipidemia refers to abnormally elevated levels of lipids and/or lipoproteins in the blood, indicating a defect in lipoprotein metabolism. It can manifest as increased cholesterol (below 200 mg/d), increased triglycerides (TG) (below 150 mg/dL), increased low-density lipoprotein cholesterol (LDL) (below 100 mg/dL), and decreased high-density lipoprotein cholesterol (HDL) (above 60 mg/dL). Controlled blood pressure refers to blood pressure that is effectively managed by antihypertensive medications (such as angiotensin-converting enzyme inhibitors, beta-blockers, diuretics, and calcium channel blockers) and non-pharmacological treatments. In this case, systolic blood pressure (SBP) is maintained below 140 mmHg, and diastolic blood pressure (DBP) is maintained below 90 mmHg. Uncontrolled or poorly controlled blood pressure indicates blood pressure that remains elevated despite the prescribed antihypertensive drugs. In this case, SBP equals or exceeds 140 mmHg, and/or DBP is 90 mmHg or higher. Anthropometric measurements are various aspects of the human body and its parts, providing quantitative indices of their variability. These indicators include height, weight, BMI, waist circumference (WC), and waist-to-hip ratio (WHR).

The article "Blood Parameter Profiles and Their Clinical Implications in Hypertensive Patients: A Retrospective Chart Review" was retracted in 2025. Reasons: errors in the data; errors in the methods; errors in the results or conclusions; errors in the images.

Statistical analyses

The SPSS version 28.0 software was employed for all statistical analyses. A significance level of p-value <0.05 was considered to indicate statistical significance. The statistical analysis included calculating descriptive statistics for age, weight, and height, stratified by gender, to explore gender differences in these variables. Additionally, for hematological parameters such as hematocrit (HCT), platelets, hemoglobin, calcium, phosphorus, sodium, potassium, urea, creatinine, and uric acid levels, mean, median, SD, and the minimum and maximum values were computed. Furthermore, a Pearson's correlation matrix was constructed to assess the relationships between these hematological parameters and demographic variables. Additionally, to compare these variables in terms of gender, an independent samples t-test was utilized. The results of these analyses are detailed in the Results section of this study.

Ethical consideration

The study obtained ethical approval from King Khalid University's local Institutional Review Board (IRB) committee, ensuring adherence to ethical guidelines. To safeguard confidentiality and data protection, all participant information was securely stored in a password-protected cloud. We strictly followed the Helsinki guidelines and ensured the anonymity of the data collection process.

## Results

Descriptive statistics for age, weight, and height of patients with HTN have been stratified by gender. For age, the mean and standard deviation are 58.65 and 13.06 for males, respectively, and 68.09 and 15.72 for females. In terms of weight, males have a mean of 77.91 with a standard deviation of 14.01, while females have a mean of 73.19 and a standard deviation of 23.63. Regarding height, the mean for males is 162.98 with a standard deviation of 8.52, whereas, for females, the mean is 154.74 with a standard deviation of 6.81. These statistics underscore the gender differences in these three variables, offering valuable insights for researchers and clinicians exploring gender-related health disparities (Table 1).

**Table 1:** Descriptive statistics for demographic characteristics of the study population.

Variables	Gender	N	Mean	SD
Age	Male	98	58.65	13.06
	Female	23	68.09	15.72
Weight	Male	96	77.91	14.01
	Female	23	73.19	23.63
Height	Male	95	162.98	8.52
	Female	23	154.74	6.81

For patients with HTN, various blood parameters were analyzed, including hemoglobin (HB), platelets, HCT, calcium, phosphorus, sodium, potassium, urea, creatinine, and uric acid. The results provided each parameter's mean, median, SD, minimum, and maximum values. According to the results, the median hemoglobin value is 14.56, with an SD of 2.27, a minimum of 8.36, and a maximum of 18.73. The mean hemoglobin value is 14.50. Similarly, the median platelets value is 250.00, with an SD of 132.76, a minimum value of 14.50, and a maximum value of 905.80. The mean platelets value is 280.99. Additionally, the median hematocrit value is 44.06, with an SD of 18.39, a minimum of 13.28, and a maximum of 215.70. The mean hematocrit value is 45.59.

The article "Blood Parameter Profiles and Their Clinical Implications in Hypertensive Patients: A Retrospective Chart Review" was retracted in 2025. Reasons: errors in the data; errors in the methods; errors in the results or conclusions; errors in the images.

Additionally, for calcium, the median value is 4.82, the mean is 5.07, the standard deviation (SD) is 1.26, and the range is 2.07-12.39. For phosphide, the median is 3.36, the mean is 3.27, and the SD is 0.88, with values ranging from 0.50 to 5.97. For sodium, the median is 136.00, the mean is 134.54, the SD is 12.99, and the range is 2.41-158.00. Further, for potassium, the median value is 4.17, the mean is 4.13, the SD is 0.48, and the range is 2.29 to 5.16. For urea, the median is 37.10, the mean is 43.88, and the SD is 27.76, with values between 9.82 and 163.95. For creatinine, the median is 1.05, the mean is 1.12, and the SD is 0.41, with the lowest value being 0.44 and the highest 3.10. For uric acid, the median is 6.16, the mean is 6.29, and the SD is 2.00, ranging from 2.75 to 13.82 (Table 2).

**Table 2:** Descriptive statistics for various blood test results. HB: Hemoglobin; HCT: Hematocrit.

Parameters	Mean	Median	SD	Minimum	Maximum
HB	14.50	14.56	2.27	8.36	18.73
Platelets	280.99	250.00	132.76	14.50	905.80
HCT	45.59	44.06	18.39	13.28	215.70
Calcium	5.07	4.82	1.26	2.07	12.39
Phosphide	3.27	3.36	.88	0.50	5.97
Sodium	134.54	136.00	12.99	2.41	158.00
Potassium	4.13	4.17	0.48	2.29	5.16
Urea	43.88	37.10	27.76	9.82	163.95
Creatinine	1.12	1.05	0.41	0.44	3.10
Uric acid	6.29	6.16	2.00	2.75	13.82

It is crucial to remember that the typical ranges for these blood parameters can vary depending on factors such as age, gender, and geographical location. Because of this, it is essential to interpret these values in light of the pertinent reference ranges. In order to investigate the connections between the 10 important variables of patients suffering from HTN, a correlation matrix was computed. There were significant positive correlations between platelets and urea (r = 0.400, p <0.01) and creatinine (r =0.517, p <0.01), as shown in the matrix. HCT and calcium also had a highly significant positive correlation (r = 0.394, p < 0.01). The correlations between HB and uric acid, HCT and uric acid, and HCT and platelets were all significantly negative (r = -0.179, p <0.05), as were the correlations between HCT and platelets (r = -0.081, p <0.05). Additionally, there were highly significant negative correlations between calcium and HB (r = -0.066, p <0.05) and calcium and platelets (r = -0.171, p <0.05). Additionally, there was a significant positive correlation between potassium and phosphate (r =0.186, p <0.05) as well as between phosphate and calcium (r =0.202, p <0.05). Finally, all the variables, except for sodium, showed statistically significant positive correlations with urea (Table 3).

The article "Blood Parameter Profiles and Their Clinical Implications in Hypertensive Patients: A Retrospective Chart Review" was retracted in 2025. Reasons: errors in the data; errors in the methods; errors in the results or conclusions; errors in the images.

**Table 3:** Correlation among various blood test results. HCT: Hematocrit, the normal hematocrit for men is 40-54%; for women it is 36-48%; HB: Hemoglobin, male: 13.8 to 17.2 grams per decilitre (g/dL), female: 12.1 to 15.1 g/dL; Normal calcium is 9-10.5 mg/dL; Normal potassium: 3.5-5.2 mEq/L; Normal phosphorus is between 3 and 4.5 mg/d; Normal result creatinine is 0.7-1.3 mg/dL ** p<0.01 (two-tailed), * p<0.05 (two-tailed).

Parameters	Uric acid	Sodium	HB	Platelets	HCT	Calcium	Phosphate	Potassium	Urea	Creatinine
Uric acid	--									
Sodium	0.058	--								
HB	-0.179	0.081	--							
Platelets	0.400^**^	-0.049	-0.203^*^	--						
HCT	-0.039	0.010	0.394^**^	-0.081	--					
Calcium	0.052	-0.050	-0.066	-0.171	0.094	--				
phosphate	0.090	-0.002	0.077	0.202^*^	0.014	-0.037	--			
potassium	0.139	0.113	0.010	0.047	-0.003	0.113	0.186	--		
Urea	0.628^**^	-0.006	-0.311^**^	0.395^**^	-0.200^*^	0.023	0.222^*^	0.250^**^	--	
Creatinine	0.517^**^	0.047	-0.214^*^	0.328^**^	-0.091	0.052	0.266^**^	0.149	0.700^**^	--

There were no discernible differences between male and female patients suffering from HTN in terms of their levels of platelets, uric acid, sodium, potassium, or urea when we compared the mean values of these variables by gender. Males had higher mean HB levels than females, though there was a significant difference (t(119) = 2.144, p =0.034). Males had higher mean creatinine levels than females, which was also a significant difference (t(119) = 2.228, p =0.008). The results show that there may be gender differences in some hematological parameters but not in others and strong correlations between some variables that should be considered in future analyses (Table 4).

**Table 4:** Mean difference between male and female in terms of various blood test results. HB: Hemoglobin; HCT: Hematocrit.

Measures	Gender	N	Mean	SD	t	P-value
HB	Male	98	14.71	2.28	2.144	0.034
	Female	23	13.60	2.07		
Platelets	Male	98	281.00	139.77	0.001	0.999
	Female	23	280.95	100.04		
HCT	Male	97	44.43	8.56	-1.425	0.157
	Female	23	50.48	38.45		
Uric Acid	Male	95	6.29	2.05	-0.009	0.993
	Female	22	6.30	1.83		
Calcium	Male	80	4.99	1.09	-1.271	0.207
	Female	20	5.39	1.79		
Phosphate	Male	79	3.30	0.77	0.719	0.474
	Female	18	3.13	1.29		
Sodium	Male	98	135.36	4.53	1.434	0.154
	Female	23	131.06	28.53		
Potassium	Male	98	4.13	0.47	0.065	0.949
	Female	23	4.12	0.55		
Urea	Male	97	43.36	27.16	-0.424	0.673
	Female	22	46.15	30.87		
Creatinine	Male	98	1.16	0.42	2.228	0.008
	Female	23	0.95	0.30		

The article "Blood Parameter Profiles and Their Clinical Implications in Hypertensive Patients: A Retrospective Chart Review" was retracted in 2025. Reasons: errors in the data; errors in the methods; errors in the results or conclusions; errors in the images.

## Discussion

The findings of this study on the hematological parameter of hypertensive patients in the region of Saudi Arabia offer essential knowledge on several parameters, including HB, platelets, HCT, calcium, phosphorus, sodium, potassium, urea, creatinine, and uric acid. To fully comprehend the implications of these findings, discussing and interpreting them in the context of earlier research on the subject is crucial. First, the study provides median and mean values for HB, platelets, and HCT, the minimum and maximum values for each, and the corresponding SDs. These factors are crucial for assessing the patient's general well-being and their risk factors for HTN. Similar results from earlier studies in Saudi Arabia have suggested that people with HTN frequently have different hematological parameters [10,11]. Age, gender, and lifestyle choices are a few variables that may impact these variations [12-14]. The study also provides information on the levels of calcium, phosphorus, sodium, and potassium, which are crucial electrolytes involved in various physiological processes, including blood pressure control. According to prior research conducted in the Saudi Arabia region, patients with HTN may experience electrolyte imbalances, which could contribute to the development or exacerbation of the condition [12,13]. Therefore, for HTN to be effectively managed, it is essential to comprehend these values and their potential effects on the condition. The study also provides values for urea, creatinine, and uric acid, which are critical indicators for evaluating kidney function. Prior studies in Saudi Arabia have shown that people with HTN are more likely to experience kidney complications [10,14]. In order to identify potential kidney dysfunction and provide the necessary interventions to stop further complications, clinicians can benefit from monitoring these parameters. It is crucial to keep in mind that these hematological parameters' normal ranges can vary depending on factors like age, gender, and location. Interpreting these values in light of the relevant reference ranges is crucial. The findings from this investigation into the hematological parameters of Saudi Arabian patients with HTN provide crucial insights into various facets of their health. These results align with prior research on HTN and its associated hematological parameters in the region. Clinicians and researchers should consider these findings when devising interventions for the effective management of HTN and its complications. Further research is needed to delve deeper into the root causes of these variations, which will enable the development of more targeted strategies to address them.

The article "Blood Parameter Profiles and Their Clinical Implications in Hypertensive Patients: A Retrospective Chart Review" was retracted in 2025. Reasons: errors in the data; errors in the methods; errors in the results or conclusions; errors in the images.

In examining the relationships between 10 essential variables for HTN patients in the Saudi Arabia region, we gain important insights into the correlations among these parameters. Discussing and interpreting these findings in the context of earlier research on the subject is crucial to better comprehending them. First, the study shows that platelets have significant positive correlations with urea and creatinine. This finding raises the possibility that kidney function and platelet levels are related in hypertensive patients. Prior studies conducted in Saudi Arabia suggested that people with HTN may be more susceptible to complications relating to the kidneys [10,15]. Thus, it is essential to comprehend these relationships to effectively manage HTN and its complications. This result aligns with prior research that showed calcium is necessary for maintaining healthy blood cell function, including creating RBCs [16,17]. The study also reported a significant negative correlation between HB and uric acid, HCT and uric acid, and HCT and platelets. These findings point to potential inverse relationships between these parameters, which in patients with HTN may indicate underlying health problems or complications. More research is required to better comprehend the clinical implications of these negative correlations and create targeted interventions to address them. The study also identifies highly significant negative correlations between calcium, platelets, and HB. These results might point to a possible calcium metabolism imbalance, which might have an impact on blood cell function and lead to the onset or worsening of HTN [12,18]. Furthermore, both phosphate and calcium, as well as potassium, exhibit strong positive correlations in the results. These correlations suggest interactions between electrolytes, which are essential for many physiological processes, including blood pressure control [13,19]. Finally, all variables, with the exception of sodium and urea, have statistically significant positive correlations. This finding emphasizes the potential value of urea as a marker for evaluating general health in hypertensive patients. The findings of this study on the correlations between critical parameters of patients with HTN in Saudi Arabia offer significant new understandings of the correlation between these parameters. These findings should be considered by clinicians and researchers when developing interventions to manage HTN and its related complications effectively. To develop focused strategies to address them, more research is required to understand the underlying causes of these correlations better. Researchers and clinicians can benefit greatly from the findings of this study on gender differences in hematological parameters among hypertensive patients in Saudi Arabia. Discussing and interpreting these findings in light of prior literature on this subject is crucial when comparing the mean values of these variables by gender while also connecting the paragraphs for better comprehension. First, the findings show no appreciable differences in platelet, uric acid, sodium, potassium, or urea levels between male and female patients with HTN. This finding is in line with some earlier local research studies that found no discernible gender differences in these parameters among hypertensive patients [11,20]. Therefore, these results imply that changes in these hematological parameters in response to HTN may be similar for both male and female patients.

The article "Blood Parameter Profiles and Their Clinical Implications in Hypertensive Patients: A Retrospective Chart Review" was retracted in 2025. Reasons: errors in the data; errors in the methods; errors in the results or conclusions; errors in the images.

The study found that males have significantly higher mean HB levels than females (t(119) = 2.144, p =0.034). This outcome is in line with earlier research that discovered gender differences in HB levels in several populations, including Saudi Arabia [17,18]. Differences in HB levels between males and females may be influenced by hormones, iron status, genetics, and other factors [16,17]. Healthcare professionals must therefore consider these gender differences when treating hypertensive patients. The results show that males also have significantly higher mean creatinine levels than females (t(119) = 2.228, p =0.008). This outcome is in line with earlier studies that demonstrated that males typically have higher levels of creatinine than females due to elements like muscle mass and kidney function [10,14]. These variations in creatinine levels must therefore be taken into account when assessing kidney function in hypertensive patients.

Based on the findings of this study, there are notable differences in height, weight, and age between the genders among HTN patients in the Saudi Arabian region. To properly discuss and interpret these results, it's essential to reference earlier research. To start, the average age of male patients with HTN is 58.65 years (SD = 13.06), while female patients average 68.09 years (SD = 15.72). Previous research conducted in Saudi Arabia suggests that women are more likely than men to develop HTN later in life [20,21]. Moreover, the average weight for male patients is 77.91 kg (SD: 14.01), while female patients average 73.19 kg (SD: 23.63). This aligns with prior research on obesity in Saudi Arabia, indicating that hypertensive men in the study population tend to be heavier than women [22,23]. Furthermore, the mean height for male patients stands at 162.98 cm (SD = 8.52), in contrast to 154.74 cm (SD = 6.81) for female patients. Given that men are generally taller than women, this difference in height is anticipated. Although taller individuals might have a reduced risk, height can still influence the likelihood of developing HTN [24].

The article "Blood Parameter Profiles and Their Clinical Implications in Hypertensive Patients: A Retrospective Chart Review" was retracted in 2025. Reasons: errors in the data; errors in the methods; errors in the results or conclusions; errors in the images.

Strengths and limitations

Despite offering insightful data, this study has some drawbacks. The sample size might not be sufficient to extrapolate the results to Saudi Arabia's entire population. Additionally, because the study is cross-sectional, it is difficult to prove that one variable causes another. Additionally, the study does not take into account possible confounding variables, such as comorbidities or medication use, which might affect the relationships that were found.

## Conclusions

This study provides valuable insights into the blood parameters of hypertensive patients in Saudi Arabia, offering information on their overall health status and potential risk factors for HTN. The research highlights the importance of considering age, gender, and lifestyle choices when managing HTN and underscores the significance of electrolyte balance and kidney function markers. The findings align with earlier studies and emphasize the need for further research to fully comprehend the underlying factors influencing these blood parameters' variations and correlations. Clinicians and researchers should consider these results when designing interventions for efficient HTN management and associated complications. Future research should focus on understanding the relationships between blood parameters, gender differences, and HTN onset in Saudi Arabia. Large-scale longitudinal studies are recommended to gain deeper insights while also exploring the impact of confounding factors like comorbidities, medications, and lifestyle choices.
